This article has been retracted.

# Comparative Expression Profile of miRNA and mRNA in Primary Peripheral Blood Mononuclear Cells Infected with Human Immunodeficiency Virus (HIV-1)

**DOI:** 10.1371/journal.pone.0022730

**Published:** 2011-07-28

**Authors:** Ankit Gupta, Pruthvi Nagilla, Hai-Son Le, Coulton Bunney, Courtney Zych, Anbupalam Thalamuthu, Ziv Bar-Joseph, Sinnakaruppan Mathavan, Velpandi Ayyavoo

**Affiliations:** 1 Department of Infectious Diseases and Microbiology, Graduate School of Public Health, University of Pittsburgh, Pittsburgh, Pennsylvania, United States of America; 2 Department of Machine Learning, Carnegie Mellon University, Pittsburgh, Pennsylvania, United States of America; 3 Human Genetics, Genome Institute of Singapore, Singapore; INSERM, France

## Abstract

Host cells respond to exogenous infectious agents such as viruses, including HIV-1. Studies have evaluated the changes associated with virus infection at the transcriptional and translational levels of the cellular genes involved in specific pathways. While this approach is useful, in our view it provides only a partial view of genome-wide changes. Recently, technological advances in the expression profiling at the microRNA (miRNA) and mRNA levels have made it possible to evaluate the changes in the components of multiple pathways. To understand the role of miRNA and its interplay with host cellular gene expression (mRNA) during HIV-1 infection, we performed a comparative global miRNA and mRNA microarray using human PBMCs infected with HIV-1. The PBMCs were derived from multiple donors and were infected with virus generated from the molecular clone pNL4-3. The results showed that HIV-1 infection led to altered regulation of 21 miRNAs and 444 mRNA more than 2-fold, with a statistical significance of p<0.05. Furthermore, the differentially regulated miRNA and mRNA were shown to be associated with host cellular pathways involved in cell cycle/proliferation, apoptosis, T-cell signaling, and immune activation. We also observed a number of inverse correlations of miRNA and mRNA expression in infected PBMCs, further confirming the interrelationship between miRNA and mRNA regulation during HIV-1 infection. These results for the first time provide evidence that the miRNA profile could be an early indicator of host cellular dysfunction induced by HIV-1.

## Introduction

There is remarkable variation in the onset of disease in HIV-1 infected individuals. The replication, spread, and immune evasion of the virus and the progression of disease depend on host cellular transcription and gene regulation in virus-specific target cells and immune cells [1], [2], [3]. Both viral and host cellular factors have been shown to contribute to infection, virus replication, and disease progression. Viral factors include free-extracellular (cell- and virus-free), virion-associated, and infected cell-associated viral antigens, as well as infectious and noninfectious virus particles. HIV-1 virus with defective expression of viral proteins such as Nef, Vpr, Gag, and Pol are shown to induce differential gene expression [4], [5], [6]. Host factors include host genetics (determined by HLA alleles), polymorphisms in HIV receptors and coreceptors, and genes involved in innate and adaptive immune responses [7], [8], [9], [10]. Following the landmark discovery of the *CCR5*-Δ32 mutation that protects against HIV infection [11], [12], [13], many other genetic variants have been shown to affect HIV infection and AIDS pathogenesis [7], [14], [15]. It is likely that, in addition to incomplete immunological control, host genetic variation and differences in gene expression in the infected host cells may also contribute to the differential disease pattern [16], [17], [18]. Along these lines, attempts were made to identify host cellular proteins associated with HIV-1 infection [19], [20], [21], [22]. There is limited information, however, regarding the regulation of host cellular genes at the transcriptional, post-transcriptional, and translational levels.

Several studies have shown that HIV-1 infection differentially regulates host cellular genes and pathways, suggesting that differential gene expression in infected individuals either accelerates disease progression or enhances resistance to the development of disease [23], [24], [25]. Genome-wide association studies have not fully defined the resistance in exposed uninfected sex workers or elite controllers, indicating a role for other host cellular factors [26]. Studies delineating the cellular factors in individuals who remain uninfected despite repeated exposures to the virus have found that they over-express anti-viral innate factors, such as RANTES, SLPI, and other chemokines [27]. It is important to note that the differential expression of host cellular genes is not universal, resulting in disease progression at variable rates in infected individuals [28], [29], [30].

Gene expression in general is regulated at transcriptional, post-transcriptional, and translational levels. Recent discoveries have emphasized a central role for the new class of small non-coding RNA in gene expression controlling growth, development, and immune response *in vivo* [31], [32], [33]. These non-coding RNAs, which include microRNA (miRNA), partition function for interacting RNA (piRNA), and small interfering RNA (siRNA), are emerging as a major component of the cellular regulatory pathways that underlie the development and physiology of complex organisms [34], [35], [36]. Regulation of gene expression by miRNA occurs primarily at the post-transcriptional level [37], [38]. Recent studies have shown that miRNA have a unique expression profile in cells of the innate and adaptive immune systems, CNS, and cancers [39], [40], [41], [42]. Based on these observations, we suggest that pathogens including viruses could potentially modulate host cellular transcription at multiple levels by targeting various factors including miRNAs.

Studies previously have evaluated the expression of either miRNA or mRNA in cells isolated from HIV-1 infected subjects [43], [44], [45], [46]. Their results are likely to be influenced by variabilities in host genetics and viral heterogeneity in addition to other factors including viral burden. In an effort to understand host cellular gene regulation during HIV-1 infection, we performed a comparative global miRNA and mRNA microarray profiling in PBMCs derived from multiple donors upon infection with HIV-1. Our results indicate that HIV-1 infection differentially regulated several miRNAs that could potentially regulate host cellular pathways such as cell cycle, apoptosis, T cell signaling and cytokine/chemokine responses. Taken together, these results for the first time provide evidence that the miRNA profile could be an early indicator of HIV-1 induced host cellular dysfunction.

## Materials and Methods

### Generation of infectious HIV-1

The infectious HIV-1 particles were generated by using the proviral DNA construct pNL4-3 obtained from the National Institutes of Health AIDS Research and Reference Reagent Program (NIH AIDS RRRP). Two million HEK293T cells (a kind gift from Dr. Michelle Calos, Stanford University) were transfected with 5 µg of proviral DNA using Polyjet (SignaGen) as suggested by the manufacturer. Virus titer was measured by p24 antigen ELISA, and infectivity was assessed by determining multiplicity of infection (MOI) using the HIV-1 reporter cell line TZM-bl (NIH AIDS RRRP) as described earlier [47].

### Isolation and infection of PBMCs with HIV-1 virus

We purchased normal donor blood from the American Red Cross Blood Bank in Pittsburgh using appropriate IRB approval forms from the University of Pittsburgh. PBMCs were isolated by Ficoll-Hypaque gradient centrifugation. Freshly isolated normal donor PBMCs (5×10^6^/mL) were stimulated with 5 µg/ml PHA-P (Sigma, St. Louis, MO) for three days. Cells were washed, divided into two parts and cultured in RPMI medium (GIBCO, CA) containing 10% FBS (Hyclone, Logan, UT), 1% L-glutamine (Cambrex, MD), 1% penicillin-streptomycin (GIBCO, CA), and IL-2 (200 U/mL, Chiron, Emoryville, CA). One half of the cells were subsequently infected with 0.1 MOI of virus particles using standard protocols as described [48] and the remaining half of the culture is maintained under similar conditions and used as control. Seven days post infection (pi), culture supernatants were assessed by p24 ELISA for infection and virus replication [47]. Cells were collected and frozen for miRNA and mRNA isolation. We performed a total of 16 independent experiments using donor PBMCs (n = 16).

### Total and miRNA isolation

PBMCs (both infected and control) were collected, washed with PBS, and lysed for RNA isolation. Total RNA was isolated using the TRIzol method (InVitrogen) as suggested by the manufacturer. Next, to enhance the sensitivity and detection, we enriched the small RNA using a microRNA isolation kit (SABiosciences) with two separating columns as per the manufacturer's instructions. This allowed us to isolate both miRNA and mRNA, which were used in the miRNA array and gene expression arrays, respectively. RNA quality was determined by chip-based capillary electrophoresis using Agilent Bioanalyzer 2100 (Agilent, CA), according to the manufacturer's instructions.

### MiRNA profiling using RT^2^ MicroRNA PCR Array

For miRNA profiling studies, we used the SABiosciences RT^2^ MicroRNA PCR Array system, an optimized real-time PCR assay, which allows the simultaneous detection of 704 miRNAs, representing most functional miRNAs, as well as appropriate housekeeping assays and RNA quality controls. We performed the assay according to the manufacturer's protocol. Enriched miRNA was converted to cDNA using an miRNA first strand synthesis kit. First strand was used to perform the miRNA PCR array using a Taqman 7900HT machine. Equal amounts of RNA from both infected and uninfected cells were used for the first strand and assayed as per the manufacturer's protocol.

### Gene expression profiling

For total mRNA profiling, we used the Illumina HT-12 array, which targets more than 25,000 annotated genes with more than 48,000 probes covering well-characterized genes, gene candidates, and splice variants. One µg of high-quality total RNA from each sample was used to generate cDNA. Sample labeling, hybridization, and scanning were performed according to the manufacturer's protocols as well as standardized protocols developed by the core laboratory at the University of Pittsburgh. Data analysis was performed using the Illumina software to delineate the false discovery rate (FDR) and differences with statistical significance (p<0.05).

### Microarray data analysis

We analyzed the expression of individual miRNA using CT values obtained with a threshold of 0.2. Endogenous controls, RT negative controls, and genomic DNA contamination controls were tested for each array. If a particular miRNA in either the control or the experiment samples showed expression at least three times with a value of 35 or greater, it was excluded from the analysis as undetectable or undetermined. We uploaded values (CT) that passed through these stringent criteria into the SABiosciences software (RT^2^ Profiler PCR Array Data Analysis) and calculated fold change for each miRNA. Data were further subjected to statistical analysis using the manufacturer's web-based software to define the difference with significant p value (p< = 0.05) between the two groups.

### Validation of differentially regulated miRNA and mRNA from the genome-wide array

Based on the data analyses, selected miRNA and mRNA targets were verified by qRT-PCR using specific primers and probes (Applied Biosystems). We used RNA samples (n = 6) from the miRNA microarray profiling to validate the high throughput microarray results. Additional validation was performed by infecting under similar conditions normal donor PBMCs (n = 10) that were not part of the miRNA microarray.

### Computational analysis validating the miRNA targets and mRNAs

To identify mRNA targets of miRNAs in the samples, we used GenMIR++ [49], a novel regression-based Bayesian method developed to identify targets of miRNAs by integrating the measured expression data for miRNAs and mRNAs with a database of a potential set of mRNA targets for each miRNA. GenMIR++ takes into account the downregulation of target mRNAs by modeling the expression of each targeted mRNA as a negatively weighted sum of the expressions of multiple miRNAs with some additional Gaussian noise. The method restricts the set of possible targets for each miRNA to a set of candidate mRNAs given *a priori*. This potential set of targets for each miRNA is derived based on sequence analysis. For this paper, we used predictions from the MicroCosm Targets database [50] to determine this set. For the GenMIR++ analysis, we first used the R package samr [51] to detect differentially expressed mRNAs by using an FDR cutoff of 10%. We next combined these mRNAs with the differentially expressed miRNAs, leading to 2,941 mRNAs and 327 miRNAs that were used as input to GenMIR++. The plots show the top 10% of interactions predicted by GenMIR++ ranked by their p-values.

### Pathway analysis

To determine gene interactions and correlation networks, we used Ingenuity Pathway Analysis, STRING, and KEGG. The cutoff values for inclusion in these analyses were differential gene expression, with p-value <0.05 and 2.0 in fold change (based on SAM). Genes identified from miRNA-based predicted targets (score of >70) were also assessed to define the potential networks and pathways.

## Results

### Infection and miRNA and mRNA quality from PBMC from multiple donors

The goal of our study was to analyze the potential link between miRNA and mRNA in HIV-1 infected cells. We hypothesized that infection of target cells such as PBMCs by HIV-1 may lead to the following scenarios: i) The infection may regulate an identical subset of miRNA in cells derived from genetically diverse individuals, and ii) The changes in miRNA may have an impact on mRNA in genes associated with distinct cellular pathways.

We used PBMCs from multiple donors to validate the differential regulation of miRNA and mRNA profiles by HIV-1 infection. All the donors were healthy and seronegative for HIV-1. To eliminate variability with regard to the virus, we used a well-characterized virus derived from a molecular clone. Infectivity was assessed by qRT-PCR using HIV-1 Gag-specific primers and probes as described [52] employing an equal amount of RNA. The presence of Gag was determined by normalizing with endogenous control and presented as CT values (Figure 1A). Samples with low and high CT values (<12 or >30) were eliminated from further profiling studies (Higher CT value (>30) indicate inefficient virus replication and lower CT value (<12) indicate high infectivity and infection induced cell death). Results indicate that infected cultures of PBMCs showed the presence of Gag with an average CT value of 21.88±1.12, indicating virus replication. Gag CT value was below the level of detection in the uninfected control. Cell death was assessed in the infected and uninfected cultures before RNA isolation (Figure 1B). Cell death in uninfected cultures ranged from 0 to 27% (an average of 8.4±2.2%), whereas infected cultures showed a higher percentage (16–50%, with an average of 29.33±2.4%). To ensure RNA quality, infected cultures with high cell death (>50%) were not included in microarray analysis.

**Figure 1:** Infectivity in and cell death in PBMCs used for analyses. **(A)** Normal donor PBMCs were infected with HIV-1 or mock infected for seven days. RNA was isolated and tested for Gag by RT-PCR. Gag CT values were obtained by using the endogenous control for normalization. Figure shows average CT value from 16 independent donors. **(B)** After seven days, post-infection cell death was assessed by trypan blue dye exclusion method. Dot blot represents percentage of cell death in uninfected (NT) and infected (HIV-1) PBMCs from 16 independent donors.

RNA isolated from these cultures was tested for quality by spectrophotometry and by Taqman assays for endogenous control miRNAs and mRNA species. Each sample was tested for two miRNA and two small RNA controls (Table 1). All but two donors showed CT values (>30) for endogenous controls. These two donors were eliminated from further analyses to avoid bias because the quality of RNA in these samples may not have been ideal for qRT-PCR profiling.

**Table 1:** Selected endogenous controls and their Ct values.

Endogenous controls	Control #1	Control #2	Control #3	Control #4	Control #5	Average
SNORD48/RNU48/U48	25.49	25.07	26.8	25.8	24.65	25.56
SNORD47/U47	19.27	21.37	19.52	21.32	22.47	20.79
SNORD44/U44	17	18.9	17.64	19.77	22.69	19.2
RNU6-2/U6-2	20.82	22.35	20.84	21.16	23.35	21.70

Endogenous controls	HIV-1#1	HIV-1 #2	HIV-1 #3	HIV-1 #4	HIV-1 #5	Average
SNORD48/RNU48/U48	20.31	24.46	27.57	23.16	25.49	24.198
SNORD47/U47	19.48	17.83	20.72	19.45	24.7	20.436
SNORD44/U44	18.97	15.69	18.53	19.17	21.67	18.806
RNU6-2/U6-2	17.82	18.35	21.35	19.57	24.37	20.292

RNA isolated from infected and uninfected PBMCs was evaluated first for the level of endogenous controls by RT-PCR using specific primers and probes as a measure of RNA quality and quantity before microarray analysis. Five representative donors out of 16 donors are presented here.

### HIV infection differentially regulated expression of multiple miRNAs

The expression profile of 704 host cellular miRNAs was assessed in infected and uninfected PBMCs from multiple donors (n = 6). Results revealed that HIV-1 infection differentially regulated expression of several miRNAs (Tables S1 and S2). The level of expression in infected cells was compared with that in uninfected cells, and fold differences were calculated based on normalization with internal controls. The fold differences ranged between 2- and 88-fold for different miRNAs. Among the total 704 miRNAs tested, 208 were upregulated (Table S1) by more than 2-fold compared to controls, and 14 were downregulated (Table S2) compared to controls. Further analyses indicated that among these 222 miRNAs, 41 were upregulated (>4-fold) and five were downregulated (>4-fold).

To further assess the significance of our data, we performed statistical analyses to identify the regulated miRNA in the infected and the uninfected groups, using 2-fold as the cutoff (Figure 2; Table 2). Results indicate that among the 208 upregulated miRNAs, 21 exhibited significant changes across multiple donors (p value of <0.05). It is interesting to note that none of the 14 miRNAs that showed downregulation exhibited significant p value. Heatmap analyses further cluster the miRNA species between the test groups (Figure 2). Together these results indicate that fold differences did not necessarily correlate with the differential regulation of miRNAs in multiple donors.

**Figure 2:** Heatmap and hierarchical clustering of miRNA. The heatmap represents the result of the two-way hierarchical clustering of miRNA and samples. Each row represents miRNA, and each column represents samples tested. The clustering is represented for the miRNA and samples on top and sides, respectively. Red represents miRNA with an expression level above the mean, and green represents miRNA with an expression level below mean/average.

**Table 2:** Significantly regulated miRNAs in HIV-1 infected cultures compared to uninfected control cells.

Mature ID	Fold change	p value	^#^Predicted targets	Cellular function based on predicted targets through TargetScan and IPA analysis
miR-593	2.3247	0.0010	67	Amino acid Metabolism
miR-431	4.2845	0.009372	25	Cell growth and proliferation
miR-892a	2.4136	0.013	122	Cellular function and Maintenance
miR-138	2.1364	0.013	44	Cell Morphology
miR-564	4.8795	0.0130 79	7	N/A
miR-628-3p	4.6012	0.017119	60	Cell Signaling
miR-411	8.2454	0.018815	29	Cell Cycle
miR-518f*	3.3215	0.0308	10	DNA Replication, Recombination and Repair
miR-187	2.0631	0.035	4	N/A
miR-188-5p	6.1813	0.037526	72	Cell Cycle
miR-938	3.6903	0.0399	15	Cellular Development
miR-1253	3.1465	0.0419	106	Cellular function and Maintenance
miR-1470	3.317	0.0425	2	N/A
miR-549	5.3005	0.04538	60	Cell Cycle
miR-888*	4.8503	0.0469	153	Cellular function and Maintenance
miR-33b*	2.9726	0.0484	79	Cellular Assembly and Organization
miR-519b-5p	2.8366	0.050	50	Nucleic acid Metabolism
miR-302a	3.6139	0.050	164	DNA Replication, Recombination and Repair
miR-1286	3.3554	0.0523	34	Carbohydrate Metabolism
miR-636	2.5808	0.0548	47	Cell Cycle
miR-760	2.9002	0.0575	42	Cell Signaling

This table lists miRNAs that are significantly regulated (over expressed) with a significance of p<0.05 in HIV-1 infected cultures compared to uninfected control cells. ^#^ Column represents targets identified through miRDB having a target score ≥70.

Based on these analyses, we selected the differentially regulated miRNAs with significant p value (<0.05) for further analyses. To understand the significance of these miRNAs in host cellular functions, we identified target genes using TargetScan followed by IPA analysis (Table 2). Our results indicate that HIV-1 infection targets cellular genes primarily involved in cell cycle, proliferation, cellular movement and migration, and cell signaling. Previous studies have reported findings that virus infection and viral antigens modulate these host cellular pathways [53], [54].

### Validation of miRNA expression by qRT-PCR

To validate the differentially regulated miRNAs from the microarray results, we randomly selected the nine miRNAs from Table 2 (miRNA with 2-fold change and p<0.05) and the five miRNAs from Tables S1 and S2 (miRNA with 2-fold increase but p>0.05). We tested RNA from the infected and uninfected control pair from multiple donor PBMCs for specific miRNA along with endogenous controls using miRNA specific primers and probes by qRT-PCR (Figure 3). Results indicate that among the nine upregulated miRNAs tested from Table 2, all except miR-628-3p showed upregulation by independent qRT-PCR assay. Although miR-628-3p showed upregulation in miRNA profiling, all donors used in independent validation did not show significant upregulation, thus resulting in no change. This could be due to variations within donors or due to design of primer/probes used in qRT-PCR. Similarly, the single downregulated miRNA, miR-120, showed downregulation in most of the tested samples. This was validated in both the samples that were used to perform the genome-wide microarray (n = 6) and additional PBMCs (n = 10) infected in a similar manner, suggesting that these miRNAs are consistently regulated across multiple donors. Validation of miRNA in both the samples further confirms that the array analyses in our samples are reproducible.

**Figure 3:** Quantitative real time RCR (qRT-PCR) confirmation of randomly selected miRNAs from the microarray analysis. The expression of selected miRNAs in PBMCs infected with HIV-1 along with the expression of uninfected controls were tested for validation by qRT-PCR using a specific primer and probe for each miRNA. Fold increase/decrease was calculated based on endogenous control normalization. Average fold change for each miRNA represents fold change obtained from 10 independent donors.

### HIV-1 induced gene regulation of cellular mRNA transcripts

miRNAs regulate cellular gene expression at the post-transcriptional level, thus silencing and/or downregulating gene expression [55], [56]. To assess whether a direct correlation exists between the expression patterns of miRNA and mRNA, we assessed the expression profile of mRNA transcripts present in HIV-1 infected PBMCs and in uninfected control cells from the same donor. Microarray profiling of mRNA samples was normalized with the internal endogenous control and cross-compared between the two groups.

Among the 48,000 transcripts tested, we found that 444 genes were differentially regulated in the infected culture compared to uninfected controls. Of the 444 differentially regulated genes, 147 were upregulated and 297 were downregulated significantly (FDR corrected with p value of <0.05 with 2-fold regulation). We analyzed these mRNA transcripts to identify the pathways using STRING, IPA, and DAVID databases. To further analyze the interplay between the up- and downregulated mRNA, all the differentially regulated mRNA were combined and evaluated. The results, which are presented in Figure 4, indicate that HIV-1 infection regulates three major clusters including SRC kinases, MAPK, and apoptosis/cell cycle regulators. Similar results were reported by previous studies using transcriptome analysis in HIV-1 infected target cells [45], [46]. Results presented in Figure 4 include both upregulated and downregulated genes. To understand whether HIV-1 targets specific pathways for up- or downregulation, we performed individual pathway analyses (Table 3 & 4). Results from the upregulated genes include clusters of genes that control cell cycle, apoptosis, DNA damage pathways, and several signaling pathways including MAPK, p53, TRL, and T-cell receptor (Table 3). In contrast, analyses of downregulated gene clusters include primarily anti-apoptotic proteins/pathways, NF-kB mediated immune dysregulation, and SRC kinases (Table 4). Additional analyses using various software and databases yielded similar results (data not shown). Collectively, these results indicate that several pathways are regulated by HIV-1 infection including inflammatory response, cell death, cell-to-cell signaling and interaction, and immune function.

**Figure 4:** Predicted interaction networks of genes regulated during HIV-1 infection. Differentially regulated genes are represented in the links predicted using STRING (http://string.embl.de/). Predicted interactions represent both direct and indirect associations that are derived from four different sources: genomic context, high throughput experiments, conserved co-expression, and previous findings from the literature. The nature of the supporting evidence is indicated by the color lines: green represents neighborhood; red, gene fusion; blue, co-occurrence; black, co-expression; purple, previous experiments; turquoise, database; yellow, text mining; and aqua, homology.

**Table 3:** Genes upregulated in the HIV-1 infected culture compared to uninfected control cells, determined by transcriptome analysis.

Canonical Pathways	Count	p Value	Genes
MAPK signaling	6	1.30E-05	PPP3CC; CACNA1I; PPP3CB; PRKCA; TGFBR2; CDC25B
T-cell receptor signaling	4	5.29E-05	MALT1; PPP3CC; PPP3CB; PRKCQ
Natural killer cell mediated cytotoxicity	4	1.32E-04	PPP3CC; PPP3CB; PRKCA; HCST
Wnt signaling	4	1.91E-04	WNT7A; PPP3CC; PPP3CB; PRKCA
Calcium signaling	4	3.96E-04	PPP3CC; CACNA1I; PPP3CB; PRKCA
B-cell receptor signaling	3	3.78E-04	MALT1; PPP3CC; PPP3CB
Long-term potentiation	3	3.78E-04	PPP3CC; PPP3CB; PRKCA
VEGF signaling	3	3.93E-04	PPP3CC; PPP3CB; PRKCA
Apoptosis	3	6.24E-04	PPP3CC; PPP3CB; ATM
Cell cycle	3	0.00144	CDC14B; ATM; CDC25B
Tight junction	3	0.00211	CLDN18; PRKCA; PRKCQ

**Table 4:** Genes downregulated in the HIV-1 infected culture compared to uninfected control cells determined by transcriptome analysis.

Pathways	#	p Value	Gene
Cell cycle	10	1.80E-10	MCM2; MCM7; PKMYT1; CDK2; GADD45B; MAD2L2; TFDP1; GADD45A; PCNA; ORC1L
Apoptosis	8	7.26E-09	IRAK2; NFKBIA; BCL2L1; TNFRSF10B; BAX; DFFA; EXOG; TNF
Purine metabolism	8	4.74E-07	ADA; ADCY3; ADCY8; POLA1; POLR3K; POLE2; GART; DGUOK
MAPK signaling	8	3.71E-05	MAP3K8; GADD45B; DUSP2; ATF4; GADD45A; DUSP5; TNF; DUSP10
Cytokine-cytokine receptor interaction	7	1.92E-04	TNFSF9; TNFRSF10B; CD70; IL8; TNF; TNFRSF18; TNFSF13B
DNA polymerase	5	5.76E-07	MCM2; MCM7; POLA1; PCNA; POLE2
Base excision repair	5	5.76E-07	PARP2; PCNA; POLE2; APEX2; POLB
Adipocytokine signaling	5	1.32E-05	SOCS3; NFKBIA; TNF; NFKBIE; CPT1A
p53 signaling	5	1.52E-05	CDK2; GADD45B; TNFRSF10B; BAX; GADD45A
Epithelial cell signaling in H.pylori infection	5	1.63E-05	NFKBIA; LYN; IL8; JAM2; SRC
Small cell lung cancer	5	4.44E-05	NFKBIA; BCL2L1; CDK2; TRAF3; TRAF4
Toll-like receptor signaling	5	1.00E-04	NFKBIA; MAP3K8; IL8; TNF; TRAF3
One carbon pool by folate	4	6.80E-07	SHMT2; GART; MTHFS; MTHFD1L
Urea cycle andmetabolism of amino groups	4	7.33E-06	ASS1; ACY1; ALDH7A1; SMS
Aminoacyl-tRNA biosynthesis	4	3.46E-05	WARS; YARS; GARS; RARS
Glycine, serine and threonine metabolism	4	4.19E-05	CBS; PHGDH; SHMT2; GARS
Gap junction	4	8.33E-04	ADCY3; ADCY8; CSNK1D; SRC
Pyrimidine metabolism	4	8.33E-04	UPP1; POLA1; POLR3K; POLE2
GnRH signaling	4	0.00140	ADCY3; ADCY8; ATF4; SRC
T cell receptor signaling	4	0.00150	NFKBIA; MAP3K8; TNF; NFKBIE
Tight junction	4	0.00335	CGN; MYL2; JAM2; SRC
Insulin signaling	4	0.00353	TRIP10; SOCS3; PFKM; PTPN1
Mismatch repair	3	1.46E-04	MSH6; PCNA; EXO1
Arginine and proline metabolism	3	5.66E-04	ASS1; PYCR1; RARS
Nucleotide excision repair	3	0.00102	ERCC1; PCNA; POLE2
Fatty acid metabolism	3	0.00109	ACADVL; ALDH7A1; CPT1A
Glutathione metabolism	3	0.00148	GSTA4; GGCT; SMS
Inositol phosphate metabolism	3	0.001952	IMPA2; INPP1; ITPKA
Amyotrophic lateral sclerosis	3	0.002056	BCL2L1; BAX; TNF
Hedgehog signaling	3	0.002163	CSNK1E; CSNK1D; RAB23
Glycolysis/Gluconeogenesis	3	0.003010	ALDH7A1; PFKM; GCK
Drug metabolism cytochrom.p450	3	0.00419	GSTA4; FMO4; CYP3A5
B-cell receptor signaling	3	0.0047	NFKBIA; LYN; NFKBIE
Chronic myeloid leukemia	3	0.0047	NFKBIA; BCL2L1; STAT5A
Phosphatidylinositol signaling	3	0.0048	IMPA2; INPP1; ITPKA
Prostate cancer	3	0.0073	NFKBIA; CDK2; ATF4
NK cell mediated cytotoxicity	3	0.0243	TNFRSF10B; ULBP1; TNF
Jak-STAT signaling	3	0.0327	SOCS3; BCL2L1; STAT5A
Calcium signaling	3	0.0501	ADCY3; ADCY8; ITPKA
Focal adhesion	3	0.0649	MYL2; SRC; PARVB

### Computational analysis validating the miRNA targets and mRNAs

Gene expression is regulated at the transcriptional and the post-transcriptional levels. A single miRNA can potentially regulate multiple mRNA; the opposite is also possible [57]. To further validate whether the observed expression profile of mRNA is directly and/or indirectly regulated by miRNA, we performed a comprehensive computational analysis of mRNA and miRNA expression profiles in HIV-1 infected samples as well as in the uninfected controls. The log ratio of infected to control for both mRNA and miRNA was normalized as suggested by the manufacturers' software (Illumina and SABiosciences) to eliminate the false discovery rate and statistical significance across multiple samples. We used the Significance Analysis of Microarray (SAM) [51] and identified 2,941 differentially expressed genes (mRNAs), which we retained for further studies.

Next, we used GenMIR++ [49] to integrate mRNA, miRNA, and sequence-based predictions into an miRNA-mRNA interaction graph (Figure 5A). GenMIR++ uses predicted miRNA targets (Methods) to generate an initial binary interaction matrix for interactions between miRNA and mRNA (Table 5). Based on this table, a linear Gaussian regression model is created for each mRNA by regressing it on the best subset of miRNAs that can potentially interact with it. Coefficients are constrained to be negative to indicate the anti-correlation between miRNAs and their targets. Using this method, we identified the top 275 interactions involving 196 mRNAs and 118 miRNAs and organized them to represent the set of interactions predicted in this dataset (Figure 5A). The results show several clusters of miRNA-mRNA regulation. For example, miR-144, miR-937, miR-376, miR-519, and miR-548A-3P are shown to regulate a number of mRNAs, and HCK, NFKBIE, IL6, SHMT2, and MCM4 are regulated by several miRNAs.

**Figure 5:** Network of predicted miRNA-mRNA interactions. **(A)** Regression-based method was used to predict the miRNAs (green circles) that are actively regulating mRNAs (red diamonds) in our dataset. **(B&C)** Validation of miRNA-mRNA interaction partners by RT-PCR using independent samples (n = 6) for IL-1ß(B) and IL-6 (C).

**Table 5:** Interplay between miRNA and mRNA based on GenMIR ++ analysis.

miRNA	Potential targets (mRNA)
let-7d*	APP, CKS1B, DDIT4, IL3RA, NFKBIA, PLSCR1
miR-129-3p	KIFC1, NAPSB, ORC1L
miR-130a	C13ORF18, DLL1, G0S2, GADD45B, STX11, TNF, TNFAIP6
miR-139-5p	BATF, KIF1A, RFC3
miR-144	BARD1, BTG3, CEP55, IDH2, IL6, KHDRBS3, LYN, SGOL1, TRIP6, ZC3H12A
miR-193a-5p	ERN1, HCK, SEMA7A, SHMT2
miR-196b	ADFP, LOR, MCM4
miR-198	CBS, COL9A2, DYSF
miR-214	MCM4, SLC11A1, TMPRSS6
miR-301b	DLL1, RAB34, SLC43A2, TFP1
miR-302c	FAIM3, IGF1R, PPA1, RSBN1L
miR-33a	ABCA1, INDO, PLTP, RAB9A, SAT1
miR-376a	C15ORF48, IL6, MMP7, TFP1, TNFAIP6
miR-501-3p	C1ORF57, NFKBIE, SASH1, TIMELESS
miR-502-3p	CATSPER1, DTX1, IL17F, SP140
miR-515-5p	ENPP3, EXO1, FANCG, HES1, MTHFD1L, POLA2
miR-517a	BARD1, GNL3, PTGES, RAD54L
miR-518c	KIFC1, NFKBIE, RBBP8, WARS
miR-518d-3p	KIFC1, MCM2, NFKBIE
miR-519e	CD9, CDC2L5, CYB561D2, EBI2, FBP1, MGAT4A, NINJ2, NPL, PYHIN1, RBL2, SORL1, TBC1D10C, TREM2
miR-520g	MCM3, MCM4, MTHFD1L, POLQ, UHRF1
miR-526b	ACADVL, OIP5, OXCT2, SLC43A3
miR-532-3p	CD70, KIFC1, SLC1A5
miR-548a-3p	ANKRD57, MEP1A, POLE2, RAD51AP1, RBBP8, SMPDL3A, TYMS
miR-548b-3p	C13ORF18, CD70, DUSP5, IER5, IL1B, KYNU, TMEM106C, WBP5
miR-548d-3p	CBS, CD70, DUSP5, GNA11, IL1B, KYNU, L2HGDH, PRPF19, IL6
miR-627	TEX264, TRIM47, TXNIP
miR-632	ASF1B, C17ORF53, DOK3, DYSF,
miR-648	AHI1, BCAR3, HELLS, TK1
miR-659	CXXC5, SHMT2, TRO
miR-744	BID, BRSK1, COL9A2
miR-920	BLR1, CDH1, RBPMS2
miR-935	IER3, MND1, PIF1, SHMT2
miR-937	C15ORF48, CABLES1, FHOD1, GADD45G, GNA15, NEU4, PLEKHA4
miR-938	CDCA5, IRF8, TYMS

These miRNAs were selected on the basis that they target at least three mRNAs with the score of >0.50001.

To validate the predicted target and miRNA combinations, we selected two miRNA-mRNA interaction clusters and assessed the level of their expression in multiple donor samples (n = 7). We selected IL-1ß and IL-6, which were upregulated in the HIV-1 infected culture but not in the uninfected control (Figure 5B). Several studies indicate that these two molecules are known to be upregulated by HIV-1 infection under similar conditions [58], [59], [60], although the role of miRNAs in regulating these cytokines is not well defined. Our interaction analyses indicate that IL-1ß could potentially be regulated by miR-211, miR-578, and miR-548d-5p. Results indicate that the expression of IL-1ß mRNA is upregulated by HIV-1 infection by 12.81±6.05-fold, whereas miR-578 is upregulated by 2.0±0.4-fold, miR-548d-5p does not show any change (Figure 5B), and miR-211 is downregulated by 4.2±0.2-fold. This indicate that among the three miRNAs tested, one showed a significant negative correlation, one showed no change, and one exhibited positive correlation. We also tested the IL-6 mRNA-miRNA interaction (Figure 5C), and results indicate a partial confirmation of the predicted results. Together, results from these confirmation analyses indicate 60–70% validation of the predicted negative correlation of miRNA and mRNA expression.

## Discussion

Previous studies have performed comparative global profiling of either mRNA or miRNA using HIV-1 infected cells and lymphoid tissue [1], [44], [61], [62], [63]. This is the first study to measure the miRNA and mRNA expression profile at the same time point in PBMCs infected with the HIV-1 virus, with the exception of one study that assessed miRNA and mRNA profiling in brain tissues from infected individuals with dementia [64]. The *in vitro* PBMC culture system that we used offers several advantages over the use of cells or tissues derived from HIV-1 infected individuals. The *in vitro* system allows analysis of miRNA and mRNA at precise points after virus infection. It also enables the use of a virus derived from proviral DNA. In combination with the ability to carry out studies using cells from multiple donors, these features may help to identify potential signature patterns with respect to the regulation of gene expression associated with virus infection.

We identified a number of significantly regulated miRNAs and mRNAs in infected PBMCs compared to uninfected control cells. Among the 704 miRNAs tested, 21 are differentially regulated with statistical significance of <0.05 p value, suggesting that virus infection does alter the miRNA expression profile. It is important to note that the significantly regulated miRNAs showed upregulation ranging from 2.1- to 8.2-fold. Although HIV-1 infection differentially regulated certain miRNAs to a higher degree (>22–88-fold), they did not show statistical significance across multiple donors.

It is worth noting that we did not observe any miRNA that is significantly downregulated by virus infection, whereas Houzet et al. [44] reported downregulation of a number of miRNAs in HIV-1 infected PBMCs obtained from HIV-1 positive subjects. It is not clear whether this difference is due to the assay platforms used, the number of miRNAs assessed, or the methodologies used to evaluate the statistical significance. It is also possible that infection level or viral load/burden could influence the level of miRNA expression. The patient population in the Houzet et al. study had relatively low viral loads compared to the *in vitro* infected cultures. Our results are in line with those from the study by Tatro et al. [64], which reported the dysregulation of miRNA in brain tissue from HIV-1 positive patients compared to that in uninfected control brain tissue. The authors reported that, of the 19 miRNAs that were dysregulated in HIV-1 positive brain tissue compared to uninfected brain tissue, six were also dysregulated in HIV-1 infected PBMCs compared to uninfected cells. They also identified brain-tissue-specific miRNAs, suggesting that their levels in PBMCs may be undetectable or tissue specific as reported before [65], [66].

Given that many pathogens including viruses depend on host cellular machinery for their replication, survival, and immune evasion, the hypothesis that particular viruses alter cellular miRNAs may not come as a surprise. Many viruses including herpes virus, Epstein-Barr virus, HCV, HHV-8, and retroviruses are known to affect host cellular miRNAs [67], [68], [69]. It is not clear, however, whether all these viruses regulate specific miRNAs for replication, immune evasion, and/or immortalization. Searching the literature to identify the miRNAs that are differentially regulated by HCV, HBV, EVB, and herpes viruses, we found a partial overlap among these viruses. For instance, Li et al. [70] performed miRNA profiling during HBV infection and identified 13 miRNAs that are differentially regulated. When we compared these to HIV-1 mediated miRNA regulation, we found that four miRNAs were similarly altered during HIV-1 infection. We also compared the miRNA profiles in two HCV-infected hepatocyte studies [67], [70] with our results from HIV-1 infected PBMCs. We observed 33% and 40% similarity, respectively, in upregulated miRNAs between our results and those of the two studies. However, we did not observe miRNAs that were similarly downregulated in HBV, HCV, or HIV infection.

It is important to keep in mind that the expression profiles were generated by using PMBCs comprising different cell types in our study. On the other hand, the HCV-mediated miRNA profiling was assessed in hepatoma cell lines, and that for EBV-induced miRNA was performed in transformed BLCL cells [67], [68]. There might be cell-type-specific miRNA and/or altered expression level of miRNAs in different cells that could contribute to the observed differences in miRNA profiling during HCV, HIV, or EBV infection. A recent report by Wu et al. [71] provides further support that the level of miRNA expression might vary among different cell types. Collectively, these studies indicate that host cells might respond to pathogens using similar miRNAs as part of the interactions between the pathogen and the host. Conversely, it is also possible to hypothesize that viruses might target certain miRNAs as part of a general virus-host interaction to aid replication and survival. A well-defined comparative analysis is required to address this. Though this manuscript focuses on HIV-1 induced host cellular miRNAs dysregulation, HIV-1 also codes for viral miRNAs that are known to modulate host cell functions and viral transcription [72], [73], [74]. However, the interplay between the viral and host miRNAs is not well defined.

miRNAs regulate the expression of target mRNAs at the post-transcriptional level [75], [76], [77]. It is now well established that a cluster of miRNAs could regulate a single mRNA and vice versa [78], [79]. Our evaluation of the miRNA and mRNA profile (44,000 probes) from RNA isolated at the same time indicates differential regulation of a number of host cellular genes (444) with the FDR-adjusted p value of <0.05. The differentially regulated genes represent pathways including cell cycle, apoptosis, T-cell receptor signaling, DNA repair, and MAPK signaling. These results are in agreement with previously published studies using CD4+ T cells, monocytes, or macrophages infected with HIV-1 [45], [46]. Although these studies used purified specific cell types, their results indicate similar pathways, suggesting that the interaction between the virus and the target cell might trigger similar gene regulation. It is not clear whether similar genes are targeted by HIV-1 in each cell type or whether similar pathways are targeted using cell-type-specific genes. Collective information from the published studies as well as our results support the latter possibility.

A recent transcriptome-analysis study using monocytes isolated from HIV-1 patients (ART naïve and post-ART therapy) identified several innate factors as upregulated [45]; these factors were in addition to the cell proliferation, apoptotic, and signaling genes, and they were not found in our study. This discrepancy could be due to the use of different viruses. In our study, we used a CXCR4-receptor-utilizing virus (NL4-3), which primarily targets T cells. Different target cells might respond differently to the interaction between the virus and the host cell, although miRNAs that are known to regulate virus replication (e.g., miRNA-198) have been found to be commonly regulated by HIV-1 in both T and monocyte/macrophage targets [80].

In this study, to gain insight into the regulation of mRNA by miRNAs, we performed the combined miRNA and mRNA profile in HIV-1 infected PBMCs. Although previous studies have identified similar host cellular pathways regulated by HIV-1, our approach provides new information regarding their regulation at the post-transcriptional level. We observed a negative correlation between the miRNA and mRNA expression profiles, similar to the observations noted with other viral infections [81]. In conclusion, our results suggest that miRNAs play a role in regulating several host cellular genes during HIV-1 infection, altering the host cell response to the virus. Similar approaches including the role of viral load, immune activation, and HAART will provide useful information regarding biomarkers to predict disease development and the effect of HAART during early stages of the disease.

## Supporting Information

Table S1 **MicroRNAs over expressed in HIV-1 NL43 infected cultures compared to uninfected control cells.** Cut-off was 2 fold change.
(DOCX)

Table S2 **MicroRNAs under expressed in HIV-1 NL43 infected cultures compared to uninfected control cells.** Cut-off was 2-fold change.
(DOCX)
